RETRACTED

# Distribution characteristics of insect diversity in long-term fixed monitoring plots in Northeast China

**DOI:** 10.1371/journal.pone.0250689

**Published:** 2021-08-18

**Authors:** Jinwen Liu, Xiujuan Yan, Xinyuan Song, Jiamei Zhang, Donghui Wu, Meixiang Gao

**Affiliations:** 1 College of Earth Science, Jilin University, Changchun, China; 2 Jilin Academy of Agricultural Sciences, Changchun, China; 3 Northeast Institute of Geography and Agroecology, Chinese Academy of Science, Changchun, China; 4 Horticultural College of Shenyang Agriculral University, Shenyang, China; 5 Key Laboratory of Remote Sensing Monitoring of Geographic Environment, College of Heilongjiang Province, Harbin Normal University, Harbin, China; Ministry of Natural Resources North Sea Bureau, CHINA

## Abstract

The spatial patterns of field arthropod communities are an essential part of ecology and can provide fundamental data regarding field ecological processes and reveal the mechanism of ecosystem biodiversity maintenance. This study investigated the spatial distribution pattern of field insect communities to detect the spatial relationships between insect communities in farmland. The study site was located at the Dehui Agro-ecological Experimental Station of Black Soil, Jilin, China. Insect communities and environmental factors were sampled at 121 uniformly distributed points in a 400 × 400 m plot in August, September, and October 2015. The analysis revealed that insect communities from June to October demonstrated significant spatial correlation, and 6085 samples of 47 species and 47 families in 11 orders were collected from the insect community in the farmland. The farmland insect community structure changes and dynamic changes of nutritional function groups occur with time. According to the 400 x 400 m plot, the diversity of farmland insect communities and functional groups is maintained at a relatively high and stable level. In this study, a total of 6085 samples of corn farmland insects were obtained using the fluke method and direct observation method, including 11 orders, 26 families and 47 species, 4 absolute dominant populations, 6 main dominant populations, and 37 other populations. These studies can provide help for pest control in the spring corn area of Northeast China.

## Introduction

Structure and composition are important characteristics of arthropod communities. Mendenhall et al. (2014) reflected the changes of the arthropod community over time and the effect of the interaction between the plant community and arthropod community [1]. The abundance and diversity of arthropods are related to the types, structural complexity, geographic location, and environmental heterogeneity of host plants. The structure and dynamics of arthropod communities follow the characteristics of plant communities and rationally adjust the structure of biological communities where pests are located to the control effectiveness of natural enemies and the anti-insect effectiveness of host plants. This achieves continuous ecological control of pests at the community level. Mäder (2002), Bardgett (2010), and Dee (2014) project that biodiversity is a measurable characteristic of communities, and it is an index to study the level of community structure. Studies have demonstrated that diversity depends on the number and uniformity of species in the community [2–4]. It not only reflects the richness and variation of species in the community but also reflects different geographic conditions, natural environmental conditions, and community development to varying degrees. Therefore, because of the pest control strategies formulated by Johnson in 2013, it is crucial to consider the temporal changes in the richness, abundance, and diversity of arthropod species, thus becoming one of the central topics of modern ecology. Various methods of measuring diversity have also been emerging. Various calculation formulas from probability theory to information theory continue to penetrate ecology [5]. However, they are not consistent regarding various formulas and the relationship between diversity and richness, stability, and other factors. This is consistent with the diversity distribution of mayfly [6]. Because the functions of various biological species are different, it is impossible to achieve uniformity at the species level. Simultaneously, due to the lack of systematic research on the occurrence laws of farmland pests in the past, there is a certain blindness of pest control and improper control measures and pesticide abuse. While ineffectively controlling the occurrence of pests, it also violates the principle of the sustainable development of corn. To understand the occurrence law and mechanism of farmland pests more comprehensively, we systematically investigate and analyze the structure and dynamics of the arthropod community. We aim to study the problem regarding the difficulties in consistency and redefining the classification level of biological species in community research. Loreau (2001), Chang (2013), Carlander (1995), and Cardinale (2006) studied the structure and dynamics of farmland arthropod communities to explore the interrelationships between species within the community, the internal mechanism of mutual restraint, the occurrence and development of pests, pest population forecasting, and optimal control, etc. Predictions of natural enemies and integrated pest management provided a scientific basis [7–10].

RETRACTED

This research will carry out long-term systematic monitoring of corn farmland. On the one hand, it will reveal the mechanism of insect population biodiversity in farmland, the existence of farmland biodiversity allows natural control of population numbers among organisms, and on the other hand, it will provide technical support for pest control in spring corn farmland in Northeast China.

This paper researched a novel the structure, function and dynamics of farmland arthropod communities, to explore the interrelationships between species within the community. In particular, the internal mechanism of mutual restraint is researched which can come true the occurrence and development of pests, pest population forecasting and optimal control. The research of this paper is significant for the eco-control research.

The aim of the this research is to answer the following questions about a long-term monitoring plots cropfield ecosystem. (1) Does the distribution of insects show a spatial dependence, and to what extent does the distribution form a patch pattern? (2) Is this spatial distribution pattern temporal or spatial structural stability? (3) Does the reveal of the temporal and spatial distribution patterns of insect populations have a guiding effect on pest control?

## Materials and methods

### Experimental sites

The experiment was set at a permanent farmland plot (16 hm^2^) of the Dehui Agro-ecological Experimental Station of Black Soil (46° 36’ N, 125° 30’ E) of the Chinese Academy of Sciences in the central Songliao Plain of Jilin Province, China (Fig 1). The plot is in the central part of the Northeast China Spring Corn Belt and has been in the planting area for more than 50 years. The climate of the region is a temperate continental climate, with dry and cold winters and warm and humid summers. The annual average temperature is 4.4°C, and the average annual rainfall is 520 mm, of which 80% of the rainfall is concentrated in July and August. Dehui has 214,000 hm^2^ of cultivated land, of which 163,000 hm^2^ is corn, accounting for 76.2% of the total cultivated land area [11, 12].

**Fig 1:** Sixteen hectares of black soil cornfield fixed monitoring plot location. The map shows the administrative divisions of China. The solid line in the picture is northeast of China. The red dot is the location of the experiment. The shaded area is the black soil distribution area. This map was drawn by our laboratory based on the long-term experimental investigation of the approximate distribution of the black soil area in the middle of the Northeast Plain.

### Plot setting

The plot was in rectangular farmland of 500 m × 600 m and is a conventional farming field. The management of water and fertilizer farming is consistent, and herbicides are used for weeding. The terrain in the study plot is gentle, which is the most effective way to prevent the interference of the protective forest around the cornfield. The experiment site was set in the central area of the farmland to reduce the edge effect. The size of the test plot was determined to be 400 × 400 m^2^. The GPS receiver, real-time dynamic measurement, and RTK (Real Time Kinematic) measurement technology were used, and the 16 hm^2^ large square was divided into 400 20 × 20 m small squares. The test plot was divided into 441 intersections with a sampling distance of 20 m (Fig 2) [11, 12].

RETRACTED

**Fig 2:** Dimensions of sampling field. On the left is the actual distribution of farmland. The grid area in the right map shows monitoring plots with 40 m intervals, and the point (0, 0) is the coordinate origin of the monitoring graph.

### Investigation method

The sample survey was conducted from 40 × 40 m, and there were 121 intersections. The biodiversity of aphid and ant communities in Dehui’s herbicide-tolerant corn was investigated by direct observation and vacuum suction method. In this experiment, we regard the intersection as the sampling center in the field. We surveyed the right side of each point for approximately 5 months on June 1, July 6, August 1, September 2, and October 4 in five growth stages of the crops. The corn plant was directly observed and sucked by the insect sucker. After collection, the fluke bags were removed and transferred to the laboratory to identify and classify the captured insects [13].

### Evaluation model

#### Analysis of community characteristics using Raunkiaer’s frequency and coefficient of variation

Species frequency was calculated according to Raunkiaer’s formula:

Frequency = number of plots of a species in the community / total number of plots × 100%

Frequency level division standard: A: 1%~20%; B: 21%~40%; C: 41%~60%; D: 61%~80%; E:81%~100%. The frequency of Raunkiaer is A > B > C > D < E.

The coefficient of variation reflects the degree of dispersion or difference of data, namely, the distribution of data, reflecting the heterogeneous characteristics of animal data.

Coefficient of variation (CV) = standard deviation/average

The coefficient of variation reflects the degree of dispersion of the species distribution. CV < 0.1 is weak variation; 0.1 < CV < 1 is moderate variation; CV > 1 is strong variation [11].

#### Analysis of farmland insect diversity index

The statistics of spatial insect community diversity adopt the following calculation methods:

1. Relative abundance: P_i_ = N_i_/N, where N_i_ is the number of individuals of the i-th species, and N is the total number of individuals.

……………………………………………… (3.1)

2. Berger-Parker Dominance Index(D):The Berger Parker calculator returns the Berger-Parker dominance index for an OTU definition. This calculator can be used in the summary single, collect single, and rarefaction single commands.

RETRACTED

D = N_max_/N (3.2)

Nmax = the abundance of the dominant OTU

3. Shannon-Wiener Diversity index (H′):It is an index used to investigate the local biodiversity of biological communities.

H′ = -ΣP_i_lnP_i(j = 1 to s)_ (3.3)

4. Pielou Uniformity Index (J):Refers to the distribution of the number of individuals in a community or environment of all species.

J = H/H_max_ = lnS (3.4)

H_max_ is the community diversity index when a given species is completely uniform; S is the number of species.

5. Margalef Richness index (D):Refers to the ratio of the species to the number of individuals in a biological community, and is a statistic used to describe the diversity of a community.

D = (S-1)/LnN (3.5)

6. Possibility interspecies encounter:It is the chance of encounters between various groups in multiple communities.

PIE = N(N-1)/Σn_i_(N_i_-1) (3.6)

In formulas (1) to (6): N is the total number of individuals in the species; S is the number of species in the community; and n_i_ is the number of individuals in the i-th species [12].

#### Analysis of relative stability of farmland insect communities

In the experiment, the data can reflect the complexity of the relationship between the farm community food web and the natural enemies-pests and the principal component analysis of the three stability indicators constructs the community stability comprehensive index using SPSS 21.0 software.

## Result and discussion

### Composition and quantity structure of farmland insect community

According to the investigation of the whole corn growth period of the long-term fixed monitoring plot, the farmland sample specimens were classified and identified through statistical analysis (Table 1). We found that 6085 samples of 47 species and 47 families in 11 orders were collected from the insect community in the farmland. Among them, 4095 samples of 25 orders, 25 families, and 6 orders of phytophagous insects were the main farmland groups; 239 samples of 9 species, 4 families, and 3 orders were predatory insects; 2 orders, 4 families, 5 species, 540 samples were parasitic natural enemies; 4 orders, 5 families, 8 species, 1211 samples were neutral insects. Natural enemies of ladybugs and carabidae are important natural enemy groups in farmland ecosystems. Through the specific distribution of insect populations, pest control can be carried out.

RETRACTED

**Table 1:** Composition of insect community structure in corn farmland.

Species		June			July			August			September			October		
Functional group	Species		%	CV		%	CV		%	CV		%	CV		%	CV
Herbivorous insects																
Lepidoptera																
Noctuidae	*Agrotis ypcilon Rottem-berg*				6A	0.6	1.67	2A	0.1	0.71						
	*Mythimna separata Walker*				1A	0.1	2.0	16A	0.6	1.33	4A	0.3	1.06	2A	0.4	1.41
	*Spodoptera litura Fabricius*							3A	0.1	1.41	1A	0.1	1.41			
	*Helicoverpa armigera (Hübner)*							2A	0.1	1.41	4A	0.3	1.41	1A	0.2	1.41
Pyralidae	*Ostrinia furnacalis Guenée*	7A	2.0	1.50	22A	2.4	1.36	3A	0.1	0.94	2A	0.1	0.71			
Homoptera																
Cicadellidae	*Cicadella viridis*				2A	0.2	2.0	9A	0.3	1.26						
Delphacidae	*Laodelphax striatellus Fallén*				11A	1.2	1.45	266C	9.2	1.28	5A	0.3	1.13			
Aphididae	*Rhopalosiphum Maidis*	6A	1.8	1.76	281C	30.2	1.85	1362E	47.2	1.35	568E	38.6	1.37	129B	28.0	1.40
Coleoptera																
Melolonthidae	*Holotrichia diomphalia Bates*	33B	9.9	1.84	9A	1.0	1.78									
Coccinellidae	*Henosepilachna vigintioctomaculata*				7A	0.8	2.00	54B	1.9	1.31	62C	4.2	1.37	7A	1.5	1.01
Chrysomelidae	*Monolepta hieroglyphica*	4A	1.2	1.97	72A	7.7	1.44	540E	18.7	1.39	338E	22.9	1.38	71B	15.4	1.39
	*Chrysomelidae sp*.							11A	0.4	1.29	5A	0.3	1.12			
Curculionidae	*Xylinophorus mongolicus Faust*	9A	2.6	0.36	4A	0.4	1.50									
	*Sitophilus zeamais Motschulsky*															
Scarabaeidae	*Protaetia Brevitarsis*							1A	0.1	2.12	4A	0.3		11A	2.4	1.29
Rutelidae	*Anomala exoleta Fald*	2A	0.6	2.05	27A	2.9	1.85									
Elateridae	*Agriotes fuscicollis Miwa*	6A	1.8	1.32												
Hemiptera																
Pentatomidae	*Dolycoris baccarum*				2A	0.2	1.00				1A	0.1	1.41			
Pyrrhocoridae	*Pyrrhocoris sibiricus*				2A	0.2	2.00									
Miridae	*Trigonotylus ruficornis Geoffroy*							2A	0.1	0.71						
Orthoptera																
Locustidae	*Locusta migratoria manilensis Meyen*				1A	0.1	2.00	4A	0.1	1.06	6A	0.4	1.41			
Oedipodidae	*Oedaleus decorus asiaticus*							2A	0.1	1.41						
Gryllidae	*Teleogryllus infernalis*							3A	0.1	1.41	1A	0.1	1.41			
	*Teleogryllus occipitalis*							1A	0.1	2.12	1A	0.1	0.00			
Thysanoptera																
Thripidae	*Franklinielle tenuicornis Uzel*							14A	0.5	1.31	63B	4.3	1.39			
Subtotal	*4095*	67			447			2295			1065			221		
Predatory insect													0.94			
Coleoptera																
Coccinellidae	*Propylaea ajaponica Thunberg*							2A	0.1	1.41	3A	0.2		5A	1.1	1.13
	*Harmonia axyridis Pallas*	5A	1.4	1.58	3A	0.3	1.33	12A	0.4	1.18	22A	1.5	1.35	89D	19.3	1.38
	*Coccinella septempunctata Linnaeus*							3A	0.1	0.94						
Carabidae	*Amara chalcites*				3A	0.3	2.00	12A	0.4	1.06	5A	0.3	1.13	3A	0.7	0.94
	*Chlaenius bioculatus*				2A	0.2	2.00	7A	0.2	1.21	3A	0.2	0.94	2A	0.4	0.71
	*Calosoma lugens*				3A	0.3	0.67	6A	0.2	1.08	2A	0.1	1.41			
Mantodea																
Mantidae	*Tenodera Sinensls Saussure*				1A	0.1	2.00	2A	0.1	1.41						
Neuroptera																
Chrysopidae	*Chrysoperla sinica*				1A	0.1	2.00	10A	0.3	1.27	27A	1.8	1.31	4A	0.9	1.06
	*Chrysopa pallens (Ramber)*							2A	0.1	1.34						
Subtotal	*239*	5			13			56			62			103		
Parasitic insects																
Hymenoptera																
Aphidiidae	*Ephedrus plagiator Ness*							13A	0.4	1.31	82C	5.6	1.38	73C	15.8	1.36
Trichogrammatidae	*Trichogramma ostriniae Pang et Chen*				9A	1.0	1.56	6A	0.2	1.18	5A	0.3	0.85			
Ichneumonidae	*Ichneumonidae sp*.*1*							110C	3.8	1.35	63C	4.3	1.39	3A	0.7	0.94
	*Ichneumonidae sp*.*2*							57B	2.0	1.36	22A	1.5	1.29			
Diptera																
Syrphoidae	*Episyrphus balteatus De Geer*	2A	0.6	2.63	3A	0.3	1.02	51C	1.8	1.39	24B	1.6	1.30	17A	3.7	1.25
Subtotal	*540*	2			12			237			196			93		
Neutral insect																
Hymenoptera																
Formicidae	*Lasius alienus*	207D	62.2	1.98	352E	37.8	1.85	162E	5.6	1.40	95C	6.4	1.38	24A	5.2	1.24
	*Camponotus japonicus Mayr*	16A	4.8	2.14	53B	5.7	1.94	71D	2.5	1.39	34B	2.3	1.33	12A	2.6	1.30
Diptera																
Culicidae	*Anopheles sinensis Wiedemann*	2A	0.6	1.32	25A	2.7	1.76	34C	1.2	1.25	7A	0.5	1.21			
	*Culicidae sp*.							5A	0.2	1.13	2A	0.1	1.41			
Muscidae	*Musca domestica Linnaeus*	14A	4.1	2.26	28B	3.0	0.57	8A	0.3	1.06	5A	0.3	1.13	7A	1.5	0.81
	*Calliphora vicina Robineau-Desvoidy*				1A	0.1	2.00	7A	0.2	1.21	4A	0.3	1.06	1A	0.2	1.41
Dermaptera																
Forficulina	*Dermaptera sp*.*1*							6A	0.2	1.18	3A	0.2	1.41			
Coleoptera																
Staphylinidae	*Oxytelus batiuculus*	20A	6.0	1.99				6A	0.2	0.94						
Subtotal	1211	259			459			299			150			44		
total	6085	333			931			887			1473			461		

Coefficient of variation (CV) = standard deviation/average. The coefficient of variation reflects the degree of dispersion of the species distribution. CV < 0.1 is weak variation; 0.1 < CV < 1 is moderate variation; CV > 1 is strong variation.

RETRACTED

### Farmland insect community structure changes with time

The number of species and individuals of farmland insect populations changed significantly throughout the corn growth stage (Table 1). The number of individuals per month for June, July, August, September, and October was 405, 1390, 5226, 2573, and 781, respectively, and the difference between the months was extremely significant (Fig 3) (P < 0.01), which is also related to the growth period of corn. Considering the number of species, it the largest in August, with 42 species, and least in June with 16 species. The difference between the number of species in June and July is extremely significant. The difference between July and August is extremely significant, and the difference between October and August and September is extremely significant (p < 0.01). The difference between August and September is not significant (p < 0.05)

**Fig 3:** Analysis on difference of species and individuals of insect population in farmland plots. This figure shows the significance analysis of the difference between the number of individual population months in June, July, August, September and October, and the significance analysis of the difference between the number of species months (P<0.01).

### Variation of species frequency of farm insect community

From Table 1, we can see that the farmland insect population changes significantly with the month, and the corn caterpillar ant was the dominant species in June, with its number accounting for 62.2% of the total number of samples obtained. The number and species of field insect individuals were relatively small in July, the number of corn grass aphid increased rapidly, and the number of hairy corn ants also increased. However, due to the increase in the number of species and individuals at this time, the corn grass aphids and hairy corn ants represented 30.2% and 37.8% of the population, respectively. In August, the number of corn grasshopper aphid individuals further increased, accounting for 47.2% of the total monthly catches. The number of the two-spotted tarsal worms sharply increased, and the number of hairy corn ants reduced. The predominant species in the field were *Helicoverpa* aphid and *Alalus bimaculatus* in September, which accounted for 38.6% and 22.9%, respectively. By October, the dominant species was heterochromatic ladybugs, although the population was 19.3%, the frequency distribution in the field was high. In the five study months, corn caterpillars and corn grass aphid were the dominant species. The main species were the tarsal bifocal stag beetle and ladybug in the later stage. Throughout the crop growing season, the species distribution in farmland plots changed significantly and indicated that rare species are exceedingly sensitive to seasonal changes. According to the CV of different species in each month, most species have strong temporal and spatial variability (CV > 1), and very few species have medium variation (0.1 < CV < 1), indicating that large arthropod communities on the surface are heterogenous in a horizontal direction.

### Dynamic changes of nutritional function groups of farmland insect community

Maize farmland insect communities are composed of different insect groups, and there are many kinds of them. The largest number of individuals in the artificially delineated sampling points was 1473 in August. In this experiment, the farmland insect population was divided into four functional groups according to feeding habits: herbivorous insects, predatory insects, parasitic insects, and neutral insects. Herbivorous insects are generally farmland pests, which harm the growth and development of crops and become the main constraints on agricultural production targets for prevention and control. Predatory and parasitic insects are usually natural enemies that control the number of pest population outbreaks. Neutral insects are omnivorous and corrosive insects. The composition and number of individuals of each functional group in the community are essential indicators of its stability and determine the stability of each trophic level of the food web in the farmland ecosystem. From the statistical analysis of the composition of the main functional groups of the farmland insect community in Dehui City, the results are displayed in (Figs 4 and 5), the total farmland functional group phytophagous insects accounted for approximately 70%. Corn from June to July is at the seedling and jointing stage, the nutrient growth is vigorous, and the main phytophagous insect present in this early stage is also a harmful insect.

RETRACTED

**Fig 4:** Number of individuals of farm insect functional groups changes with time. The four functional populations of insect communities in corn farmland: herbivorous insects, predatory insects, parasitic insects and neutral insects change with the month.

**Fig 5:** Farmland insect functional group species number changes with time. The four functional group species number of insect communities in corn farmland: herbivorous insects, predatory insects, parasitic insects and neutral insects change with the month.

The *Holotrichia oblita* Faldermann chafer accounted for nearly 50% of the phytophagous insects and 63% in August. The herbivorous insects accounted for nearly 80%, demonstrating that harmful insects have an absolute advantage in the entire farmland. The corn grasshopper aphid and the two-spotted tarsaled beetle accounted for 83% of the herbivorous insects. Therefore, it can be inferred that in the vigorous period of corn growth, the two herbivorous insects became the most crucial harmful population. By September and October, the two insects were still important pests, accounting for 85% and 90% of the herbivorous insects, respectively. Predatory and parasitic natural enemy insects are the main components of the natural farmland control of harmful insects.

RETRACTED

Regarding the total number, natural enemy insects can account for more than 10% of the total number of individual insects. From the perspective of individual numbers, the proportion of natural enemy insects are relatively little, but the predatory insects feed on a large quantity, such as the heterochromatic ladybug, which can prey on 3500 aphids. The parasitic efficiency of parasitic natural enemies is also extremely high and can reach 102%. Neutral insects account for 20% of farmland insects, which are mainly omnivorous or saprophytic insects. In farmland, in 2015 and 2010, Allan and Gabriel found that natural insects can regulate the relationship between harmful insects and natural enemies and eliminate the effects of farm straw and falling objects. It is also an essential functional group in farmland insect communities [14, 15].

### Ecological dominance of farmland insect community

The ecological dominance index is a measure reflecting the structural characteristics of various communities in the ecosystem. The differences in planting structure, management level, changes in land resource distribution, and phenological characteristics of farmland ecosystems have caused changes in the spatial and temporal ecological dominance index of species [16]. Therefore, the measurement of this indicator can comprehensively evaluate the dynamic changes of farmland pests and natural enemies and then use the law of dynamic occurrence of natural enemy populations to effectively control the farmland pests and provide guidance. In the farmland ecosystem, the ecological dominance index can comprehensively measure each population in the community on a quantitative level and reflect the dominance of various groups in the community according to this metric value. The more unevenly distributed the species, the more prominent the dominant population is. Conversely, it displays that if the population in the community is evenly distributed, the dominant population is occupied by multiple species. Along with the different growth periods of corn growth and the temporal and spatial changes of farmland insect communities, the ecological dominance of the main functional groups of farmland insect animal communities’ changes with the growth and development of corn (Table 2). D > 0.1 is the absolute dominant species, D > 0.01 is the main dominant species(D, Berger-Parker Dominance Index). During the entire growth period of corn, except for the low food quantity in the seedling stage in June, the herbivorous pest population has always occupied the absolute advantage status of the population. The dominance of herbivorous pests reached a maximum of 0.7510 in August, and its ecological dominance displayed a low-high-low change trend. The following and lagging effects of the natural enemy groups in each functional group are exceptionally significant. Neutral insects displayed a predominance distribution from high to low in each corn growth period. In June and July, neutral omnivorous insects, corn caterpillars, were the absolute dominant species and gradually became the main dominant population; they play an important ecological function. From the entire ecological dominance table, we can see that the functional dominance of ecological dominance varies greatly from June to August, indicating that the ecological environment of the corn farmland ecosystem is relatively simple, and able to resist human interference differences [17].

RETRACTED

**Table 2:** Ecological dominance of functional groups of farmland insect communities.

Species		June	July	August	September	October
Functional group	Food habit					
Herbivorous insects	Harmful insects	0.3498	0.3927	0.6369	0.5466	0.6163
Predatory insect	Natural enemies	0.0150	0.0097	0.0118	0.0333	0.1931
Parasitic insect	Natural enemies	0.0060	0.1794	0.0381	0.1147	0.1952
Neutral insects	Omnivorous or corrosive	0.6216	0.3781	0.0925	0.0876	0.0781

Berger-Parker Dominance Index(D), The Berger Parker calculator returns the Berger-Parker dominance index for an OTU definition. This calculator can be used in the summary single, collect single, and rarefaction single commands. D > 0.1 is the absolute dominant species, D > 0.01 is the main dominant species.

### Farmland insect community biodiversity distribution

In 2010, Christoph believed that the diversity of species was the key to biodiversity. It not only embodied the complex relationship between organisms and the environment but also embodied the richness of biological resources [18]. Diversity not only reflects the richness and variability of the community but also reflects the relationship between different natural geographic conditions and community development to varying degrees. One of the characteristics of the stability of biological communities is high diversity. It is one of the central topics of modern ecology research. The farmland ecosystem is an ecosystem under human interference. The diversity of farmland insect and animal communities is not only related to the number of species, population ratio, interspecies relationships, and the complexity of the food web but also closely related to the growth and development stages of corn and human factors [19]. Table 3 demonstrates that the structural trends of farmland diversity are quite unstable because the farmland has a single planting structure, all of which are corn. This only provides a place for insects that feed on corn, and the structure of species biodiversity is simple. Therefore, maize farmland is prone to large-scale outbreaks of pests, and the population of certain dominant species is high, which leads to the instability of the community structure and the decline of diversity. In general, the management level of farmland is relatively high, and the occurrence of pests has been controlled within a certain range. Therefore, Jangid (2011) put forward that the diversity of farmland insect communities and functional groups was maintained at a relatively high and relatively stable level [20].

RETRACTED

**Table 3:** Biodiversity characteristics of farmland insect community functional groups.

Species	June			July			August			September			October		
Functional group	Shannon index	Pielou index	Margale index	Shannon index	Pielou index	Margale index	Shannon index	Pielou index	Margale index	Shannon index	Pielou index	Margale index	Shannon index	Pielou index	Margale index
Herbivorous insects	0.7412	0.4624	0.7198	0.7953	0.4941	0.6526	1.3307	0.6399	1.2280	1.1146	0.5728	1.1975	1.0634	0.7671	0.7928
Predatory insect	-	-	-	1.6977	0.9475	1.9494	1.9809	0.9015	1.9874	1.3366	0.7459	1.2115	0.5788	0.3596	0.8631
Parasitic insect	1.8181	1.8181	1.4270	1.4875	1.4413	2.1303	1.6659	1.4640	2.1968	1.8556	1.8468	2.0084	1.6899	1.6899	0.9262
Neutral insects	0.7442	0.4624	0.7198	0.7953	0.4941	0.6526	1.3307	0.6399	1.2280	1.1146	0.5728	1.1975	1.0634	0.7671	0.7928
All populations	1.5045	0.5701	2.2338	1.8824	0.5711	3.8033	1.9101	0.5178	4.8945	2.0917	0.5983	4.3865	2.0703	0.7163	2.7717

Shannon-Wiener Diversity index, it is an index used to investigate the local biodiversity of biological communities. Pielou Uniformity Index, refers to the distribution of the number of individuals in a community or environment of all species. Margalef Richness index, refers to the ratio of the species to the number of individuals in a biological community, and is a statistic used to describe the diversity of a community.

## Conclusions

This study investigated the populations of underground soil animals, surface soil animals, and above-ground space arthropods in the long-term location plots of maize farmland in the black soil region of Northeast China. Due to the problem of experimental sub-tasks, this experiment was mainly carried out on corn farmland insects. Because corn farmland is an open agricultural ecosystem, this time only one corn growth period was investigated, and the impact of natural factors and other comprehensive factors on the arthropod community could not be considered. In 2009, Fu and Zou believed that the results of the investigation may also have certain the limitations of the study. The limitation of the research is that the past farmland biodiversity research is only limited to the farmland, while neglecting the surrounding ecological environment, such as ditch weeds and shelter belts. The conclusions still need to be further enriched and improved [21]. This study preliminarily clarified the basic distribution of insects in farmland, laying the foundation for self-regulation and pest control. The study also provides an insight into this field by detecting the spatial relationships between insect communities in a farmland, and enhances our knowledge of the spatial distribution pattern of field insect communities. I think what we have learned that can be used for future research.
